The article "Fuzzy Logic-Based Machine Learning Algorithm for Cultural and Creative Product Design" was retracted in 2023. Reasons: signs of a paper mill; suspected computer-generated content; unreliable results or conclusions; concerns about the data.

# Fuzzy Logic-Based Machine Learning Algorithm for Cultural and Creative Product Design

**DOI:** 10.1155/2022/7747192

**Published:** 2022-06-09

**Authors:** Taihua Lan

**Affiliations:** College of Fine Arts, Fujian Normal University, Fuzhou, Fujian 350117, China

## Abstract

In order to effectively assist industrial designers in the color scheme design of cultural and creative products and output color schemes that meet users' image preferences, an interactive color scheme design method for cultural and creative products based on triangular fuzzy number is proposed. Through the group consistency decision based on triangular fuzzy number, an interactive genetic evolution of the color scheme population of cultural and creative products is performed to generate color schemes that satisfy the group consistency imagery preference and satisfaction, and the final selection scheme is calculated by color beauty. This paper verifies that the method can effectively integrate the imagery preferences of group users and help industrial designers to better design color schemes for cultural and creative products through the results of multiuser decision consistency.

## 1. Introduction

Cultural and creative products based on art paintings in the market are mainly divided into two categories based on a certain theme and cultural and creative products based on different artworks of a certain form [1]. For example, cultural creative products based on paintings of Van Gogh, Monet and Klimt, whose forms include functional artifacts such as mugs, mouse pads, scarves and coasters, belong to a series of cultural creative products based on a certain theme [2]. Cultural creative products based on a certain form with fixed forms, such as umbrellas and socks, with different famous paintings printed onto them [3]. To sum up, the current combination of paintings and cultural creative product carriers is rather rigid, without finding the proper entry point, not to mention the factor of personalization, which makes it difficult to win users [4].

The characteristics of cultural and creative products include shape, size, texture, material, color, graphics, and details, but aspects such as novelty style and personalized embodiment of products are not the characteristics of products, but the psychological reactions of people to products [5–7]. At the same time, design triggers emotional reactions in people, and Peter Dismert proposed five types of emotions: instrumental, aesthetic, social, surprise, and interest [8]. Cultural experiences in products are entertaining, educational, aesthetic, and creative. Entertainment refers to the relaxation of the consumer during the experience, which is an enjoyable experience; education refers to the knowledge gained during the experience, such as understanding the shape and meaning of pottery, and the production process of pottery; aesthetics refers to the pleasure of the consumer immersed in the environment of something; creativity refers to the ability to create a product that is unique and based on a personal experience [9–13]. In this paper, an interactive color scheme design method for cultural creative products based on triangular fuzzy number is proposed. The process and basic principles of interactive genetic color scheme design are investigated, and the interactive genetic evolution of the color scheme population of cultural and creative products is carried out to generate color schemes that satisfy the consistent imagery preference and satisfaction of the group, and the final selection of the scheme is calculated by color beauty, which verifies that the method can effectively integrate the imagery preference of the group users and help industrial designers through the results of consistent multiuser decision making better design color schemes for cultural and creative products [14–16].

The article "Fuzzy Logic-Based Machine Learning Algorithm for Cultural and Creative Product Design" was retracted in 2023. Reasons: signs of a paper mill; suspected computer-generated content; unreliable results or conclusions; concerns about the data.

In this paper, based on triangular fuzzy number, an interactive genetic evolution of the color scheme population of cultural and creative products is performed to generate color schemes that satisfy the group consistency imagery preference and satisfaction, and the final selection scheme is calculated by color beauty.

## 2. Related Work

CNNs have been proposed to provide a new approach to image processing and have achieved remarkable success in the field of image recognition [17]. These were created on the basis of generative adversarial networks whose training data included more than 15,000 portraits from the 14th to the 20th century, and the system automatically generated several new works until it successfully fooled specialized tests to determine whether the work was created by a human or a machine. More recently, learned existing styles and aesthetics and were able to generate their own innovative images, and experiments found that 75% of people could not distinguish whether a painting was generated by AICAN or created by the artist [18].

A key issue in image generation is how to ensure that the generated images look realistic. To this end proposed a method for learning the shape of natural image streams directly from data using generative adversarial networks, a model that automatically adjusts the output so that all edits remain as realistic as possible and all operations are represented by constrained optimization. Deep convolutional GAN were developed in to produce some highly realistic images, but currently only for specific classes, such as faces, record covers, and room interiors. Zhang et al. [19] proposed generative adversarial networks to generate images based on text descriptions only, i.e., the model first acquires text descriptions about image synthesis, second learns and captures features in the text that describe important visual information, and then uses these features to synthesize realistic images that can fool people. Nilashi et al. [20] developed a set of image-to-image conversion algorithms and later proposed the CycleGAN framework to migrate the visual style of a set of images to other images. In addition, learning-based interactive coloring methods have been proposed [21].

The article "Fuzzy Logic-Based Machine Learning Algorithm for Cultural and Creative Product Design" was retracted in 2023. Reasons: signs of a paper mill; suspected computer-generated content; unreliable results or conclusions; concerns about the data.

Although these schemes have improved the color performance, the effect is still not good. Therefore, this scheme is more important for the performance of cultural and creative design.

## 3. Fuzzy Quantification of Color Imagery Preference

The color imagery of cultural and creative products reflects the users' psychological perceptions of the products, which are often expressed with the help of language and have ambiguity and uncertainty. The triangular fuzzy number helps to solve the problem that quantitative numbers cannot fully express the evaluation opinion, so this paper introduces the triangular fuzzy number to quantify the users' color imagery preference [22–24].

Let the set of comments *I*={*i*_0_, *i*_1_, ⋯, *i*_*n*_} represent an ordered set of linguistic evaluation values, where *i*_*m*_(1 ≤ *m* ≤ *n*) is a linguistic evaluation result in this linguistic set, then the triangular fuzzy number of this result can be expressed as

(1) $$\begin{array}{c} \tilde{A}=\left(a^{L},a^{M},a^{U}\right)=\left(\frac{m-1}{n},\frac{m}{n},\frac{m+1}{n}\right). \end{array}$$

In particular, when *m* = 0, $\tilde{A}=\left(0,0,\left(m+1\right)/n\right)$.

The Likert five-level scale is used to determine the evaluation level of color imagery of cultural and creative products (*n* = 4), and the corresponding triangular fuzzy numbers and scales are shown in Table 1.

## 4. Consensus Model of Group Imagery Preference

In order to make the color scheme design of tourism cultural and creative products better reflect the image preference of users, multiple user groups are used to participate in the interactive color scheme design process. The consistency of user groups' perception of the design scheme reflects the reliability of the color scheme design results. Through interactive genetic evolution of the color scheme group of cultural and creative products, generate a color scheme that meets the image preference and satisfaction of group consistency. Therefore, we constructed a consensus model to judge the consistency of group perception [25–27].

The article "Fuzzy Logic-Based Machine Learning Algorithm for Cultural and Creative Product Design" was retracted in 2023. Reasons: signs of a paper mill; suspected computer-generated content; unreliable results or conclusions; concerns about the data.

Let the set of users be *E*={*e*_1_, *e*_2_, ⋯, *e*_*t*_}(*t* ≥ 2). According to (1) and Table 1, the triangular fuzzy number of users *e*_*i*_(1 ≤ *i* ≤ *t*) evaluating the color scheme of cultural and creative products is *a*_*i*_=(*a*_*i*_^*L*^, *a*_*i*_^*M*^, *a*_*i*_^*U*^), and the group evaluation matrix is

(2) $$\begin{array}{c} A=\left(\begin{array}{c} {\tilde{a}}_{1}\\ \vdots \\ {\tilde{a}}_{i}\\ \vdots \\ {\tilde{a}}_{t} \end{array}\right)=\left(\begin{array}{ccc} a_{1}^{L} & a_{1}^{M} & a_{1}^{U}\\ \vdots & \vdots & \vdots \\ a_{i}^{L} & a_{i}^{M} & a_{i}^{U}\\ \vdots & \vdots & \vdots \\ a_{t}^{L} & a_{t}^{M} & a_{t}^{U} \end{array}\right). \end{array}$$

The Euclidean distance is used to measure the difference of user groups' preference for color imagery of cultural and creative products, and the distance between the 2 sets of triangular fuzzy numbers *a*_*i*_=(*a*_*i*_^*L*^, *a*_*i*_^*M*^, *a*_*i*_^*U*^) and *a*_*j*_=(*a*_*j*_^*L*^, *a*_*j*_^*M*^, *a*_*j*_^*L*^) is calculated as

(3) $$\begin{array}{c} \frac{\left\|{\tilde{a}}_{i}-{\tilde{a}}_{j}\right\|=}{\sqrt{{\left(a_{i}^{L}-a_{j}^{L}\right)}^{2}+{\left(a_{i}^{M}-a_{j}^{M}\right)}^{2}+{\left(a_{i}^{U}-a_{j}^{U}\right)}^{2}}}. \end{array}$$

Then, the distance between the group evaluation matrices is

(4) $$\begin{array}{c} S=\sum_{i=1}^{t}\sum_{j=1}^{t}\left\|{\tilde{a}}_{i}-{\tilde{a}}_{j}\right\|. \end{array}$$

Using the arithmetic mean *φ* aggregates all distances as

(5) $$\begin{array}{c} B=\varphi \left(S\right). \end{array}$$

For a certain scheme of color scheme design of cultural and creative products, the consensus degree of imagery preference of user groups is

(6) $$\begin{array}{c} C_{r}=1-B. \end{array}$$

## 5. Group Consensus-Driven Interactive Color Scheme Design

### 5.1. Interactive Color Matching Design Process

Interactive genetic algorithm is an evolutionary algorithm to simulate the superiority and inferiority of biological populations, evolving color schemes through selection, crossover and variation, generating color schemes that satisfy the consistent imagery preference and satisfaction of the population, and finally obtaining a satisfactory color scheme through color beauty calculation. Compared with traditional genetic algorithm, interactive genetic algorithm adds interactive evaluation with users and embeds implicit factors such as users' preferences and perceptions into the algorithm, which can obtain a satisfactory solution more in line with users' perceptions [27]. In this paper, we consider the problem of consistency of user evaluation in the population interactive genetic algorithm, and the process of interactive genetic color matching is driven by both the consensus degree of group opinion and satisfaction based on the quantification of user imagery preference, and its color matching design process is shown in Figure 1.

The article "Fuzzy Logic-Based Machine Learning Algorithm for Cultural and Creative Product Design" was retracted in 2023. Reasons: signs of a paper mill; suspected computer-generated content; unreliable results or conclusions; concerns about the data.

### 5.2. Color Matching Interactive Genetic Manipulation

#### 5.2.1. Population Setting

The number of populations is set by the designer according to the actual demand. The individual coding method adopted in the color scheme is

(7) $$\begin{array}{c} D=\left\{\left(d_{1},r_{1},g_{1},b_{1}\right),\cdots ,\left(d_{x},r_{y},g_{y},b_{y}\right)\right\},\left(x\geq y\right), \end{array}$$

where *x* is the number of color partitions; *d*_*i*_ is the *i*-th color scheme of the product, *i* = 1, 2, ..., *x*; *y* is the number of colors included in the product color scheme; *r*_*j*_, *g*_*j*_, *b*_*j*_ is the *R*, *G*, *B* color value of a color scheme, respectively, taking values between 0 and 255 [28, 29].

#### 5.2.2. Generate the Initial Population

After obtaining the population individual code by (7), the initialized population is obtained by randomly generating the individual color by adopting the interactive genetic algorithm.

## 6. Color Beauty Calculation

In order to better reflect the quality of the output solution of interactive color scheme of cultural and creative products, color beauty is introduced to analyze the success degree of color scheme design. The color aesthetics includes the sense of order and the complexity of the color scheme, which is calculated as follows:

(8) $$\begin{array}{c} M=\frac{O}{C}, \end{array}$$

where *M* is the degree of beauty, *O* is the order factor, and *C* is the complexity factor.

The order factor *O* is calculated as follows:

(9) $$\begin{array}{c} \left\{\begin{array}{c} O=\sum O_{g}\\ O=\sum O_{h}+\sum O_{v}+\sum O_{c} \end{array}\right., \end{array}$$

where *O*_*g*_ is the order factor when only uncolored grays are combined; *O*_*h*_, *O*_*v*_, and *O*_*c*_ are the order factors determined by the color phase difference, lightness difference, and purity difference, respectively, when there are colors involved in the color scheme.

The complexity of color matching is obtained by calculating the total number of colors and the number of pairs with hue difference, lightness difference, and purity difference among all possible combinations of color pairs, thus obtaining the complexity factor C, as shown in (10).

(10) $$\begin{array}{c} C=C_{m}+C_{h}+C_{v}+C_{c}. \end{array}$$

In which, *C*_*m*_ is the total number of colors in the color scheme; *C*_*h*_ is the number of color pairs with hue difference among all possible color pairs; *C*_*v*_ is the number of color pairs with lightness difference among all possible color pairs; *C*_*c*_ is the number of color pairs with purity difference among all possible color pairs. According to (9) to (10), the color order and color complexity are calculated, and the color beauty *M* is further calculated. When *M* > 0.5, the product color scheme is considered beautiful and conforms to the law of aesthetics, otherwise it is considered unattractive.

The article "Fuzzy Logic-Based Machine Learning Algorithm for Cultural and Creative Product Design" was retracted in 2023. Reasons: signs of a paper mill; suspected computer-generated content; unreliable results or conclusions; concerns about the data.

### 6.1. Example Application Results Analysis

The cloisonné tire making is used as an innovative design example for algorithm simulation and genetic algorithm is used as a comparison. The example process finds the specific substructure of cartoon expression modeling to satisfy the target maximum group, and the execution parameters of the algorithm in this paper are shown in Table 2. The execution process of this paper is shown in Table 3, and the algorithm mining is executed 410 times.

### 6.2. Emoji Modeling Results

After reaching the target adaptation value of 0, the results of the optimized combination of cartoon expression modeling were obtained, of which the combination modeling results are shown in Figure 2. After the designer and user satisfaction survey, all the 9 cartoon expressions got 85 points (out of 100) or more, which verified the feasibility and effectiveness of the proposed method.

### 6.3. Cloisonné Making Session

The traditional cloisonné pattern making (tire making) is to cut out different shapes of purple copper sheets according to the drawings, and hammer them into various shapes of copper tires, then join the parts together and put on the solder, and after high temperature welding, they become the copper tire shape of the vessel [30].

In the process of cloisonné making, the traditional process is optimized through digital technology. Firstly, the traditional cloisonné vessels are measured and collected by laser scanning or photography to generate 3D model data of cloisonné tires, and the 3D scanning modeling is shown in Figure 3. Secondly, using deep learning and innovation engine to create 3D objects, AI achieves modeling of high-level data abstraction through image recognition technology, and deep neural network will analyze and learn from the stored traditional ware data to select 3D works that meet the requirements according to the cloisonné tire pattern specification and send them to online 3D printing platform for 3D printing. AI is useful in the model design, material selection, and product production of cloisonné 3D printing, realizing the intelligence of the whole process from design to copper tire forming. The intelligent creation of cloisonné body integrates AI with the “object,” which makes traditional craftsmen more accurate, time-saving, and labor-saving in the production of copper tires, and provides more possibilities for digital innovation design of cloisonné [31].Taking cloisonné color scheme design as an example, it is verified that the proposed method can effectively integrate the imagery preferences of group users and assist industrial designers to better design the color scheme of cultural and creative products through the results of multiuser decision consistency.

The article "Fuzzy Logic-Based Machine Learning Algorithm for Cultural and Creative Product Design" was retracted in 2023. Reasons: signs of a paper mill; suspected computer-generated content; unreliable results or conclusions; concerns about the data.

When solving iteratively with Fluent, the flow field needs to be initialized. Still, an initial velocity is added to the liquid drip inlet plane and then the solution is solved iteratively (10 iterations). After solving, the simulation results are observed and analyzed. Figures 4 and 5 show the velocity field distribution vectors obtained after the simulation.

According to the velocity field distribution obtained from the simulation, Figure 4, the velocity field distribution of the main channel shows a decreasing trend, the further away from the drip channel, the smaller the velocity vector, but the velocity field distribution exists in all areas of the main channel, and the velocity vector is distributed in the order of 10–2–10^2^ cm/s. Figure 4 shows a partial enlargement of the printhead structure, which shows that the velocity field distribution also exists in the microchamber and capillary channels, with velocity vectors in the order of 10–2 to 100 cm/s. This indicates that the velocity field distribution exists in all parts of the printhead in the presence of velocity pressure at the drip inlet [32].

## 7. Comparative Analysis of Mining Capacity

In addition, in order to evaluate the mining performance of the algorithm quantitatively, the similarity value index is used to compare the maximum cluster structure mining results of the genetic algorithm and the algorithm in this paper, and the similarity value index *S* is calculated as follows:

(11) $$\begin{array}{c} S=\frac{N_{C}}{N_{s}}, \end{array}$$

where *N*_*C*_ denotes the number of triangular slices of the largest group structure and *N*_*S*_ denotes the number of triangular slices of the template structure. The average excavation index and time comparison of the 9 cartoon expression modeling results are shown in Table 4.

As can be seen from Table 4, compared with the genetic algorithm, the algorithm in this paper consumes less time and has less similarity between structures due to the controllable execution parameters and clear objectives, thus effectively improving the design efficiency while ensuring product diversity and quality.

## 8. Conclusions

In this paper, an interactive color matching design method for cultural creative products with triangular fuzzy numbers is proposed. The user group's imagery preference is quantitatively described by using triangular fuzzy number, and the interactive genetic evolution of the color matching population of cultural creative products is operated by the group consistency decision based on the triangular fuzzy number. The proposed method is verified to be effective in integrating the imagery preferences of the group users by taking cloisonné color scheme design as an example.

The article "Fuzzy Logic-Based Machine Learning Algorithm for Cultural and Creative Product Design" was retracted in 2023. Reasons: signs of a paper mill; suspected computer-generated content; unreliable results or conclusions; concerns about the data.

## Figures and Tables

**Figure 1:** Color scheme operation flow.

**Figure 2:** Cartoon expression modeling optimization results.

**Figure 3:** 3D scanning modeling.

**Figure 4:** Micro bubble generator printhead model speed vector distribution.

**Figure 5:** Micro bubble generator printhead model velocity vector distribution (partial enlargement).

**Table 1:** Evaluation language sets.

Language evaluation variables	Triangular fuzzy number	Evaluation scale
I do not like it very much	(0, 0, 0.25)	0
Dislike	(0, 0.25, 0.5)	0.25
Commonly	(0.25, 0.5, 0.75)	0.5
Like	(0.5, 0.75, 1)	00.75
Like it very much	(0.75, 1, 1)	1

**Table 2:** Implementation parameters of this paper.

Parameter	Numerical value
Initial temperature	1000
Termination temperature	0.1
Temperature variation coefficient	0.89
Function fitness	0

**Table 3:** Implementation process of this paper.

Number of executions	Temperature	Fitness value
1	991	10
2	980.9	10
3	971.2	8
4	967.3	8
280	50.6	5
410	37.9	0

**Table 4:** Comparison of mining metrics and time.

Algorithm	Similarity (S)	Time (S)
Genetic algorithm	0.79	0.36
Simulated annealing algorithm	0.59	0.21

## Data Availability

The experimental data used to support the findings of this study are available from the corresponding author upon request.
